RETRACTED

# Noncoding RNAs and Virus and Treatment in Allergic Rhinitis

**DOI:** 10.1155/2022/1979447

**Published:** 2022-10-15

**Authors:** Zhu Lei, Guangrui Feng, Zhiguo Wang, Zhifeng Ning

**Affiliations:** ^1^Otolaryngology Department, Xianning First People's Hospital, Xianning 437100, Hubei, China; ^2^Cardiovascular Medicine Department, The First Affiliated Hospital of Hubei University of Science and Technology, Xianning 437100, Hubei, China; ^3^Dermatology Department, The First Affiliated Hospital of Hubei University of Science and Technology, Xianning 437100, Hubei, China; ^4^Human Anatomy Department, Basic Medicine College, Hubei University of Science and Technology, Xianning 437100, Hubei, China

## Abstract

Allergic rhinitis (AR) is a type I hypersensitivity reaction disease caused by inhaled allergens and immunoglobulin *E* (IgE)-mediated. Noncoding RNA (ncRNA) is an important regulator involved in gene expression and can be detected in the cytoplasm or extracellular fluid, which mainly includes microRNAs (miRNA, length 22–24 nucleotides), long noncoding RNAs (lncRNA, length >200 nucleotides), and circRNAs. LncRNA and miRNA both participate in the regulation of immune function. Some respiratory viral infections can aggravate allergic rhinitis, such as a respiratory syncytial virus (RSV) and human metapneumovirus (hMPV). However, the interaction between viral infection and allergy is complex and the mechanism is still unclear. In this review, we summarized the interactions of noncoding RNAs and viruses in the occurrence and development of AR, along with the treatments focusing on the noncoding RNAs in the past five years.

## 1. Introduction

Allergic rhinitis (AR) is a type I hypersensitivity reaction disease caused by inhaled allergens and immunoglobulin *E* (IgE)-mediated. At present, the morbidity of AR is estimated between 10% and 40% worldwide, with even up to 50% in some countries [1–3]. When allergic rhinitis patients first contact with an allergen, they never develop any clinical symptoms but have them during the sensitization stage. At this phase, dendritic cells (DCs) of the nasal mucosa take up the allergen, process it, and nest it to the draining lymph node, presenting it to the naive CD4^+^T cells [4, 5]. Subsequently, naive CD4^+^T cells are activated and differentiated into allergen-specific helper T cells type 2 (Th2 cells), which activate B cells to differentiate into plasma cells, resulting in the production of allergen-specific IgE [6–8] and release into the circulatory system. When the body is exposed to the same allergen again that can be specifically combined with IgE. This promotes effector cells' release of multiple inflammatory mediators, including histamine, leukotriene, prostaglandin D2, and other products [9].

RETRACTED

Noncoding RNA (ncRNA) is an important regulator involved in gene expression and can be detected in the cytoplasm or extracellular fluid, which mainly includes microRNAs (miRNA, length 22–24 nucleotides), long noncoding RNAs (lncRNA, length >200 nucleotides), and circRNAs [10, 11]. All ncRNA were evolutionarily conserved and coded independently [12]. LncRNA and miRNA both participate in immune regulatory responses by regulating the differentiation of bone marrow hematopoietic stem cells and activating mononuclear macrophages and DCs [13]. More interestingly, a large number of noncoding fragments were found in peripheral blood cells of patients with asthma, including natural antisense chains, pseudogenes, and differential expression of ncRNA between genes [14]. In addition, some scholars found a large number of lncRNA in CD4^+^ and CD8^+^T cells, with phased expression [15, 16]. At the same time, the role of miRNA in regulating innate immune responses, especially macrophages and granulocytes, has been shown to alter cell development, differentiation, and the release of inflammatory factors. In addition, Th2 cells are important mediators of type I allergy, and it has been reported that ncRNA promotes Th2 cell migration to target organs by regulating chemokine gene expression [17]. These results suggest that the noncoding RNA regulatory network may play a potential role in the development of allergic rhinitis (Figure 1).

Viral tinfections are known to aggravate AR. Although, the interaction between viral infection and allergy is complex and the mechanisms remain unclear. Some studies suggest that coregulatory molecules and cytokines may play a role [18]. Viral regulation of B7 family inhibitory molecules in epithelial cells leads to suppression or termination of immune responses [19]. Programmed cell death ligands 1 (PD-L1, B7–H1, CD274) and (PD-L2, B7-DC, CD273) belong to the B7 family and are widely expressed in activated T cells, B cells, monocytes, dendritic cells, macrophages, and other cells to regulate activation or inhibition [20]. NcRNA can act as a regulator of translation by participating in transcriptional and post-transcriptional gene regulation, heterochromatin formation, histone modification, DNA methylation, RNA splicing, and gene expression [21]. Many respiratory virus infections can significantly alter the expression profile of host ncRNA, and some affected ncRNA have been shown to play an important role in viral replication and/or host response [22], such as a respiratory syncytial virus (RSV) and human metapneumovirus (hMPV).

In this review, we will focus on how noncoding RNA and viruses interact to jointly regulate the occurrence and development of allergic rhinitis, as well as the latest research progress on virus-like particles and targeted noncoding RNA therapy in the treatment of allergic rhinitis patients.

RETRACTED

### 1.1. The Interaction between miRNA and Virus Copromotes the Occurrence of AR

Infectious eukaryotic viruses play an important role in acute upper respiratory tract infections. RSV and hMPV are the main viruses that cause allergic rhinitis and are also risk factors for AR [23]. These viruses cause lung injury through various immune pathways, such as activation of preinflammatory mediators (including TNF-*α*, interleukin, and chemotherapeutic factors), as well as activation of white blood cells at the infection site, resulting in impaired lung function, persistent bronchial hyperreactivity, and airway inflammation, promoting Th2 cell sensitization and inducing allergic rhinitis [24]. Microarray and high-throughput sequencing techniques have been used to identify changes in miRNA expression after RSV/hMPV infection. Changes in miRNA expression after RSV infection have been demonstrated in a variety of cells and tissues such as bronchial epithelial cells (NHBEs), nasal mucosa, and dendritic cells [25]. Members of the LEt-7 family have been shown to decrease in both animal models and human studies of asthma and allergic rhinitis. Conversely, the activation of the JAK1/STAT3 signaling pathway inhibits IL-13 production and SOCS4 gene transcription, thus inhibiting the expression of various inflammatory factors in AR. A group of core miRNAs involved in atopic diseases includes up-regulation of miR-21, MiR-223, MiR-146a, MiR-142-5p, MiR-142-3p, MiR-146b, and MiR-155 and down-regulation of let-7 family , MiR-193b and MiR-375. Most of the miRNAs involved increased Th2 cytokine secretion (MiR-124b and MiR-146b), decreased Th1 cytokine secretion (MiR-513-5p and MiR-625-5p) or promoted T cell differentiation into Th2 (MiR-21 and MiR-19a) [26, 27]. In a study of 30 patients with allergic rhinitis, we collected nasal irrigation fluid and isolated type 2 macrophages (M2) by flow cytometer. MiR-202-5p was highly expressed in macrophages of patients with allergic rhinitis compared with healthy controls, promoting M2 polarization by targeting MATN2 [28]. MiR-155 plays an important role in the development of the immune system, the differentiation of immune cells, and the maintenance of immune function. The nasal mucosa of patients with allergic rhinitis shows enrichment of ILC2 and miR-155. Highly expressed miR-155 may enhance IL-4 levels by promoting ILC2 expression, thereby promoting Th2 inflammation [29]. After RSV infection, SOCS1 and SOCS3 expressions can be induced to further reduce the phosphorylation level of STAT, which is conducive to virus survival [30]. MiR-155 and its target gene SOCS1 are key regulators of effector CD8^+^ T cells and affect cytokine signal transduction through STAT5. SOCS1 is a direct target of miR-155, and the inhibition of miR-155 can restore SOCS1 expression. Overexpression of miR-155 can reduce SOCS1 expression level [31]. Therefore, SOCS1 expression was induced after RSV infection, and the expression level of miR-155 was up-regulated. Overexpression of miR-155 can increase the surface level of IL-4 and promote the inflammatory response of allergic rhinitis patients. On the other hand, up-regulated miR-155 can inhibit RSV replication by upregulating STAT phosphorylation levels. Therefore, miR-155 can be used as a therapeutic target for patients with RSV-induced allergic rhinitis. We summarized the miRNA that plays a regulatory role in allergic rhinitis over the years (Table 1).

RETRACTED

### 1.2. LncRNA and Viruses Play Important Roles in the Occurrence of AR

Studies have found that lncRNA is associated with AR. One study showed that analysis of lncRNA cores showed that there were 2259 lncRNA in the nasal mucous membrane of AR patients, of which 1033 were up-regulated and 1226 down-regulated [38]. Genetic ontology table of enrichment results of gene ontology (GO) and pathway LncRNA-mRNA is involved in several biological processes related to the pathogenesis of AR enrichment in cell signaling pathways, such as positive regulation of IL-13 secretion and Fc*ε*RI signaling pathway and NF‐*κ*B signaling pathway [38]. Recently, it has been found that long noncoding RNA FOXD3-AS1 has a negative regulatory role in allergic rhinitis. LncFOXD3-AS1 expression in nasal mucosa was compared between patients with allergic rhinitis and healthy controls. Nasal epithelial cells (NECs) were then coincubated with lipopolysaccharide or recombinant IL-25, and NECs supernatant was then incubated with CD4+ T cells. The proportion of Th2 cells was detected by a flow cytometer. The results showed that lncFOXD3-AS1 expression was down-regulated in the nasal mucosa, and the proportion of Th2 cells in peripheral blood and the levels of IL-25, IL-4, and IL-13 were increased in AR patients, while overexpression of lncFOXD3-AS1 inhibited the expression and secretion of IL-25 in NECs, thus alleviating the inflammatory response in AR patients [39]. TNF-*α* and IL-6 are highly expressed in AR subjects and are important proinflammatory factors regulating the inflammatory response of AR. Studies have shown that their single nucleotide polymorphisms (SNPs) may be risk factors for AR susceptibility [40]. In addition, IL-6 is an inhibitor of T helper 1 (Th1) differentiation and plays an important role in regulating CD4+ T cell differentiation and IL-4 production during Th2 differentiation. Therefore, IL-6 is a key factor in regulating the pathogenesis of AR induced by the imbalance of Th1 and Th2 differentiation [41]. The research shows that down-regulated lncRNA-AK149641 can decrease the expression level of TNF-*α* and IL-6 by the activity of the NF-*κ*B signaling pathway in OVA mice [42]. We have mentioned that respiratory syncytial virus (RSV) infection is a risk factor for allergic rhinitis. Recently, some scholars found that the expression level of LncRNA-PVT1 was down-regulated in the RSV-infected AR rat model. Subsequently, we up-regulated lncRNA-PVT1 with *α*-asarone and found that the viability, proliferation, and migration of RSV-ASMCs were significantly reduced, which is mediated by the PVT1/ miR-203a/E2F3 signaling pathway [43]. These results suggest that lncrNA-PVT1 can be an important target for the prevention and treatment of RSV-induced allergic rhinitis. Finally, we concluded that LncRNA participates in the regulation and development of allergic rhinitis in recent years (Table 2).

RETRACTED

### 1.3. Recent Advances in the Treatment of Allergic Rhinitis, Focusing on ncRNA and Virus

According to the definition proposed by the ARIA (allergic rhinitis and its effects on asthma) initiative allergic rhinitis is an IgE-mediated inflammatory response of the nasal epithelium with corresponding symptoms caused by exposure to allergens [49]. Although there are many drugs to treat allergic rhinitis, many of them are symptomatic treatments, such as inhibiting histamine release or reducing inflammation, which are not the most effective ways. In addition to active allergen avoidance, immunotherapy is considered the most effective treatment for type I allergies, which includes the use of allergen agents in various forms and through various channels. Allergen immunotherapy (AIT) is the only proven effective treatment in these areas[50]. Among them, virus-like particles (VLPs) provide a very effective platform for allergen immunity, with characteristics of high immunogenicity, low allergen, and high clinical efficacy [51]. CpG motifs (CpGs) short nucleotide sequences within the CpG motif have also been extensively studied as effective stimulators of dendritic cells and B cells. The way VLPs modulate the immune response highlights its particular promise as a platform for immunotherapy of allergic diseases. Due to the immunomodulatory properties associated with viral structure, they are also used as a treatment for allergic diseases, particularly allergic rhinitis and asthma. In fact, VLPs loaded with CpGs appear to promote the re-establishment of physiological immune response in patients with allergies, although the underlying immune mechanisms are not fully understood.

RETRACTED

So how does AIT work? A dendritic cell, one of the antigen-presenting cells, is believed to play a central role in the absorption and processing of allergens to induce allergen-specific immune responses. In the presence of high doses of allergens, the physical immune system will tolerate the phenomenon, which leads to an imbalance between Th1 and Th2. Regulatory T cells (iTreg) and thymus-derived FOXP3^+^CD4^+^CD25^+^ natural regulatory T cells (nTreg) both play an important role in controlling pathogenic effector T cells and maintaining the balance between immune tolerance and immunity, which can down-regulate dendritic cells, mast cells, eosinophil and basophils, and helper T cells [52]. What's more, IL-10 and TGF-*β* are inhibitory cytokines that play an important role in this regard. When we restored the balance between Th2/Th1/Treg with VLPs, the ratio between allergen-specific IgE and IgG4 antibodies was reduced, resulting in higher IgG4 production and reduced migration of inflammatory cells to tissues, resulting in reduced clinical symptoms in AR patients.

In addition, several ncRNA-virus products are being actively developed. RNA interference (RNAi) is a gene-specific RNA degradation process mediated by short interfering RNA (siRNA), which is a novel therapeutic vector for allergic rhinitis [53]. Calcium-activated potassium ion channel-3.1 (KCa3.1) plays an important role in the release of inflammatory factors by mast cells. Some scholars investigated the effect of lentivirus-mediated shRNA silencing KCa3.1 on hypersensitivity to allergic rhinitis in mice. The results showed that LV-KCA3.1-shrNA intervention could effectively attenuate hypersensitivity to AR and inhibit mast cell activity by inhibiting PI3K/AKT signaling pathway [54]. In addition, miRNA and lncRNA both play an important role in regulating the pathogenesis of allergic inflammation, such as regulating Th1 and Th2 polarization and participating in the release of eosinophils, T cells, mast cells, and basophil cytokines. Therefore, the construction of a complete RNA regulatory network can help us better find targets for AR therapy.

## 2. Discussion

In conclusion, miRNA can target AR-related gene expression, while lncRNA can combine with miRNA through competition, and total also involved in AR epigenetic modification. On the other hand, lncRNA also may be involved in the pathogenesis of AR through multiple functional pathways. In addition, extracellular exosomes lncRNA is gaining increasing attention in AR. Further exploration of RNA in many ways will greatly expand the genes and molecules involved in the research on the mechanism of action in AR and other allergic diseases will provide the accuracy of AR in future therapy and offer new directions. Viral infections, like respiratory syncytial virus (RSV) and human metapneumovirus (hMPV), could interact with the noncoding RNA. However, the interaction between viral infection, noncoding RNA, and allergy is complex. At present, the research on allergic rhinitis is more and more in-depth, and the regulatory network of lncRNA is gradually improved, which is conducive to the development of new treatment methods and the discovery of new molecular markers for rapid diagnosis and classification.

RETRACTED

## Figures and Tables

**Figure 1:** Mechanism of allergic rhinitis. The interaction networks between ncRNA and virus copromote the occurrence of allergic rhinitis. Black arrows mark the positive effects between elements, whereas red stop bars denote inhibitory effects.

**Table 1:** Summary of regulation and function with miRNA in allergic rhinitis.

miRNA	Expression	Targets	Pathways	Function
miR-133b	Down-regulated	TNF-*α*, il-4, and INF-*α*	Nlrp3	Up-regulation of miR-133b significantly reduced OVA-specific IgE concentrations, nasal friction, sneezing frequency, cytokines (TNF-*α*, IL-4, IL-5, and IFN-*γ*), and Nlrp3 expression levels [32].
miR-181a	Up-regulated	IL-10 and TGF-*β*	PI3K/Akt	Up-regulation of miR-181a promotes expression of TGF-*β* and IL-10 and is involved in the regulation of regulatory T cell differentiation and function in children with allergic rhinitis [33].
miR-375	Up-regulated	Thymic stromal lymphopoietin (TSLP) and type II innate lymphoid cells (ILC2)	JAK2/STAT3	Mediated regulation of ILC2 cells through TSLP in allergic rhinitis [34].
miR-233	Up-regulated	IL-35		Mir-223 and IL-35 levels were associated with Th1/Th2 cytokines, eosinophil counts, and clinical severity [35].
miR-30a-5p	Up-regulated	SOCS3	SOCS1/SOCS3	Involved in T helper cell differentiation [36].
miR-202-5p	Up-regulated	CD4+T	MANT2	Promoted tregs differentiation [28].
miR-29	Down-regulated	CD276		Decreasing inflammatory response [37].

**Table 2:** Summary of regulation and function with lncRNA in allergic rhinitis.

lncRNA	Expression	Targets	Effectors	Function
Linc00632	Down-regulated	MiR-498	IL-13 and gm-csf	Linc00632 inhibited IL-13-induced GM-CSF, eotaxin, and MUAC5AC production in IL-13-treated NECs by targeting miR-498 [44].
SNHG16	Up-regulated	miR-106-5p	Leukemia inhibitory factor (LIF) and JAK1/STAT3	SNHG16 up-regulates LIF expression by binding with miR-106b-5p, thus promoting the activity of the JAK1/STAT3 pathway and promoting cell apoptosis, inflammation, and development of AR [45].
GAS5	Up-regulated	miR-140 and niR-21	IFN-*γ* and IL-2	GAS5 down-regulates the expression of target proteins, including miR-140 and miR-21, accelerates the imbalance of Th1/Th2, and promotes the inflammatory response of AR patients [46].
MIAT	Up-regulated	miR-10b-5p	Th17, IL4, IL6, and IL17	MIAT can promote allergic inflammation and symptoms by activating the th17/IL4/IL6 immune response via target-inhibited miR-10b-5p in AR patients [47].
NEAT1	Up-regulated	miR-511	NR4A2 and IL13	NEAT1 induced inflammatory cytokine production and apoptosis contributing to the pathogenesis of AR via the miR-511/NR4A2 axis [48].

RETRACTED

## Data Availability

All data in this paper are available on the PUBMED website.

## References

[1] Dinmezel S., Ogus C., Erengin H. (2005). The prevalence of asthma, allergic rhinitis, and atopy in Antalya, Turkey. *Allergy and Asthma Proceedings*.

[2] Bachert C., van Cauwenberge P., Olbrecht J. (2006). Prevalence, classification and perception of allergic and nonallergic rhinitis in Belgium. *Allergy*.

[3] Bousquet P. J., Leynaert B., Neukirch F. (2008). Geographical distribution of atopic rhinitis in the European community respiratory health survey I. *Allergy*.

[4] Humbert M., Bousquet J., Bachert C. (2019). IgE-mediated multimorbidities in allergic asthma and the potential for omalizumab therapy. *Journal of Allergy and Clinical Immunology: In Practice*.

[5] Palomares O., Akdis M., Martín-Fontecha M., Akdis C. A. (2017). Mechanisms of immune regulation in allergic diseases: the role of regulatory T and B cells. *Immunological Reviews*.

[6] Bernstein D. I., Schwartz G., Bernstein J. A. (2016). Allergic rhinitis: mechanisms and treatment. *Immunology and Allergy Clinics of North America*.

[7] Janeway C. A., Travers P., Walport M. (2001). *Immunobiology: The Immune System in Health and Disease*.

[8] Ihara F., Sakurai D., Yonekura S. (2018). Identification of specifically reduced Th2 cell subsets in allergic rhinitis patients after sublingual immunotherapy. *Allergy*.

[9] Numminen J. (2017). Allergic rhinitis. *Duodecim*.

[10] Bonnet S., Boucherat O., Paulin R. (2020). Clinical value of non-coding RNAs in cardiovascular, pulmonary, and muscle diseases. *American Journal of Physiology—Cell Physiology*.

[11] Losko M., Kotlinowski J., Jura J. (2016). Long noncoding RNAs in metabolic syndrome related disorders. *Mediators of Inflammation*.

[12] Vidigal J. A., Ventura A. (2015). The biological functions of miRNAs: lessons from in vivo studies. *Trends in Cell Biology*.

[13] Hadjicharalambous M. R., Lindsay M. A. (2019). Long non-coding RNAs and the innate immune response. *Noncoding RNA*.

RETRACTED

[14] Tsitsiou E., Williams A. E., Moschos S. A. (2012). Transcriptome analysis shows activation of circulating CD8+ T cells in patients with severe asthma. *The Journal of Allergy and Clinical Immunology*.

[15] Li M., Ma K., Feng Z., Wang J., Zhou X., Zhou L. (2020). Differential long non‑coding RNA expression profiles in the peripheral blood and CD4+ T cells of patients with active rheumatoid arthritis. *Experimental and Therapeutic Medicine*.

[16] Wells A. C., Pobezinskaya E. L., Pobezinsky L. A. (2020). Non-coding RNAs in CD8 T cell biology. *Molecular Immunology*.

[17] Zhu X. Y., Wang X. P., Wang Y., Zhao Y. (2020). Exosomal long non-coding RNA GAS5 suppresses Th1 differentiation and promotes Th2 differentiation via downregulating EZH2 and T-bet in allergic rhinitis. *Molecular Immunology*.

[18] Singh A. K., Stock P., Akbari O. (2011). Role of PD-L1 and PD-L2 in allergic diseases and asthma. *Allergy*.

[19] Ishiwata K., Watanabe N., Guo M. (2010). Costimulator B7-DC attenuates strong Th2 responses induced by *Nippostrongylus brasiliensis*. *The Journal of Immunology*.

[20] Zdrenghea M. T., Johnston S. L. (2012). Role of PD-L1/PD-1 in the immune response to respiratory viral infections. *Microbes and Infection*.

[21] Quinn J. J., Chang H. Y. (2016). Unique features of long non-coding RNA biogenesis and function. *Nature Reviews Genetics*.

[22] Wu W. Z., Choi E. J., Lee I., Lee Y. S., Bao X. (2020). Non-coding RNAs and their role in respiratory syncytial virus (RSV) and human metapneumovirus (hMPV) infections. *Viruses*.

[23] Bisgaard H., Hermansen M. N., Bonnelykke K. (2010). Association of bacteria and viruses with wheezy episodes in young children: prospective birth cohort study. *BMJ*.

[24] Rossi G. A., Colin A. A. (2015). Infantile respiratory syncytial virus and human rhinovirus infections: respective role in inception and persistence of wheezing. *European Respiratory Journal*.

[25] Wang S., Liu P., Yang P., Zheng J., Zhao D. (2017). Peripheral blood microRNAs expression is associated with infant respiratory syncytial virus infection. *Oncotarget*.

[26] Yu S. Q., Zhang R. X., Liu G. J. (2011). Microarray analysis of differentially expressed microRNAs in allergic rhinitis. *Am Journal Rhinol Allergy*.

[27] Gómez F., Rondón C., Salas M., Campo P. (2015). Local allergic rhinitis: mechanisms, diagnosis and relevance for occupational rhinitis. *Current Opinion in Allergy and Clinical Immunology*.

[28] Wang L., Liu X. Y., Song X. C., Dong L., Liu D. (2019). MiR-202-5p promotes M2 polarization in allergic rhinitis by targeting MATN2. *International Archives of Allergy and Immunology*.

RETRACTED

[29] Zhu Y. Q., Liu Y. H. (2017). A review on group 2 innate lymphoid cells and miR-155 in allergic rhinitis. *Lin Chung Er Bi Yan Hou Tou Jing Wai Ke Za Zhi*.

[30] Dudda J. C., Salaun B., Ji Y. (2013). MicroRNA-155 is required for effector CD8+ T cell responses to virus infection and cancer. *Immunity*.

[31] Wang S., Ling Y., Yao Y. Y., Zheng G., Chen W (2020). Luteolin inhibits respiratory syncytial virus replication by regulating the MiR-155/SOCS1/STAT1 signaling pathway. *Virology Journal*.

[32] Li X. F., Li J., Hu Q., Li Y. (2017). MicroRNA-133b ameliorates allergic inflammation and symptom in murine model of allergic rhinitis by targeting nlrp3. *Cellular Physiology and Biochemistry*.

[33] Zeng Q. X., Liu W. L., Luo R. Z., Lu G. (2019). MicroRNA‐181a and microRNA‐155 are involved in the regulation of the differentiation and function of regulatory T cells in allergic rhinitis children. *Pediatric Allergy and Immunology*.

[34] Luo X., zeng Q. X., Yan S. B., Liu W., Luo R. (2020). MicroRNA-375-mediated regulation of ILC2 cells through TSLP in allergic rhinitis. *World Allergy Organization Journal*.

[35] Ruan G. X., Wen X. L., Yuan Z. W. (2020). Correlation between miR-223 and IL-35 and their regulatory effect in children with allergic rhinitis. *Clinical Immunology*.

[36] Zhao C. Y., Wang W., Yao H. C., Wang X. (2018). SOCS3 is upregulated and targeted by miR30a-5p in allergic rhinitis. *International Archives of Allergy and Immunology*.

[37] Wang J., Yin J. S., Peng H., Liu A. Z. (2021). MicroRNA-29 mediates anti-inflammatory effects and alleviation of allergic responses and symptoms in mice with allergic rhinitis. *Allergy, Asthma and Clinical Immunology*.

[38] Ma Z., Teng Y., Liu X. (2017). Identification and functional profiling of differentially expressed long non-coding RNAs in nasal mucosa with allergic rhinitis. *Tohoku Journal of Experimental Medicine*.

[39] Zhang H., Zhu X. H., Liu X., Wang Y., Liu Y. (2020). Long non-coding RNA FOXD3-AS1 regulates the expression and secretion of IL-25 in nasal epithelial cells to inhibit Th2 type immunoreaction in allergic rhinitis. *Molecular and Cellular Biochemistry*.

[40] Chiang C. H., Chuang C. H., Liu S. L., Shen H. D. (2013). Genetic polymorphism of transforming growth factor *β*1 and tumor necrosis factor *α* is associated with asthma and modulates the severity of asthma. *Respiratory Care*.

[41] Lee S. Y., Bae C. S., Seo J. H. (2018). Mycoleptodonoides aitchisonii suppresses asthma via Th2 and Th1 cell regulation in an ovalbumin‑induced asthma mouse model. *Molecular Medicine Reports*.

[42] Zhang J., Zhou Y., Gu H. Y. (2020). LncRNA-AK149641 associated with airway inflammation in an OVA-induced asthma mouse model. *Journal of Bioenergetics and Biomembranes*.

RETRACTED

[43] Yu X., Zhe Z., Tang B. Q. (2017). *α*; Asarone suppresses the proliferation and migration of ASMCs through targeting the lncRNA-PVT1/miR-203a/E2F3 signal pathway in RSV-infected rats. *Acta Biochimica et Biophysica Sinica*.

[44] Yue L. Y., Yin X. Y., Hao F. (2020). Long noncoding RNA Linc00632 inhibits interleukin-13-induced inflammatory cytokine and mucus production in nasal epithelial cells. *Journal Innate Immunity*.

[45] Li H. J., Quan F., Zhang P. F., Shao Y. (2021). Long non-coding RNA SNHG16, binding with miR-106b-5p, promoted cell apoptosis and inflammation in allergic rhinitis by up-regulating leukemia inhibitory factor to activate the JAK1/STAT3 signaling pathway. *Human and Experimental Toxicology*.

[46] Song J., Wang T. J., Chen Y. D., Cen R. X. (2021). Long non‐coding RNA growth arrest‐specific 5 and its targets, microRNA‐21 and microRNA‐140, are potential biomarkers of allergic rhinitis. *Journal of Clinical Laboratory Analysis*.

[47] Ma Z. Q., Lian H. J., Lin X. Y., Li Y. (2021). LncRNA MIAT promotes allergic inflammation and symptoms by targeting MiR-10b-5p in allergic rhinitis mice. *American Journal of Rhinology and Allergy*.

[48] Wang T., Cai W. Y., Wu Q. W., Chen D., Wang P., Xu Z. (2021). Exosomal lncRNA nuclear paraspeckle assembly transcript 1 (NEAT1)contributes to the progression of allergic rhinitis via modulating microRNA-511/nuclear receptor subfamily 4 group A member 2 (NR4A2) axis. *Bioengineered*.

[49] Wise S. K., Schlosser R. J. (2012). Subcutaneous and sublingual immunotherapy for allergic rhinitis: what is the evidence. *American Journal of Rhinology and Allergy*.

[50] Calderon M. A., Gerth van Wijk R., Eichler I. (2012). Perspectives on allergen-specific immunotherapy in childhood: an EAACI position statement. *Pediatric Allergy and Immunology*.

[51] Klimek L., Kündig T., Kramer M. F. (2018). Virus-like particles (VLP) in prophylaxis and immunotherapy of allergic diseases. *Allergo Journal International*.

[52] Klimek L., Pfaar O., Bousquet J., Senti G., Kundig T. (2017). Allergen immunotherapy in allergic rhinitis: current use and future trends. *Expert Review of Clinical Immunology*.

[53] Hosoya K., Satoh T., Yamamoto Y. (2011). Gene silencing of STAT6 with siRNA ameliorates contact hypersensitivity and allergic rhinitis. *Allergy*.

[54] Lin H., Zheng C. Q., Li J., Yang C., Hu L. (2015). Lentiviral shRNA against KCa3.1 inhibits allergic response in allergic rhinitis and suppresses mast cell activity via PI3K/AKT signaling pathway. *Scientific Reports*.

